RETRACTED

# Auricular Point Pressing Beans + Continuous Intervention on *β*2-MG, Curative Effect, and Relationship with Prognosis in Elderly MHD Sufferers

**DOI:** 10.1155/2022/4166420

**Published:** 2022-09-28

**Authors:** Yan Zhou, Weiwei Cai, Xiaoxia Wang

**Affiliations:** ^1^Blood Purification Center, The Second People's Hospital Lishui, Lishui 323000, China; ^2^Second Ward, The Second People's Hospital Lishui, Lishui 323000, China

## Abstract

The effect of auricular point pressing beans + continuous intervention on *β*2-microglobulin (*β*2-MG), curative effect, and its relationship with prognosis in elderly maintenance hemodialysis (MHD) sufferers are explored. This examination selects 110 elderly MHD sufferers who are treated in our hospital from February 2020 to February 2021 as the examination objects, and they are randomly divided into two sets, 55 cases in the examination set and 55 cases in the contrast set. The sufferers in the contrast set are given routine attendance care, and the sufferers in the examination set are given auricular acupuncture combined with continuous attendance intervention. The experimental results show that for MHD sufferers, auricular acupuncture combined with continuous attendance during the therapy period can effectively enhance the clinical therapy effect, enhance the sufferers' inflammatory indexes and renal function indexes, reduce the readmission rate, and enhance the prognosis quality of life.

## 1. Introduction

Hemodialysis is a common therapy for sufferers of kidney failure. The sufferer can adjust the balance of the internal environment by replacing part of the kidney function, thereby prolonging life [1]. Due to the complexity of the disease itself and therapy, the high economic burden of maintenance hemodialysis (MHD) costs, most sufferers do not understand MHD, which leads to many negative emotions in sufferers, which seriously affects the quality of life of sufferers and health [2]. With the change in the medical model, while improving the quality of life, the quality of life of sufferers should receive more attention [3]. Attendance intervention can enable sufferers with renal failure treated with MHD to achieve the best physical, psychological and social state, eliminate negative emotions, reduce complications, enhance the MHD effect, enhance the quality of life, and prolong survival [4]. A good and high-quality continuous attendance intervention with TCM characteristics can give full play to the characteristics of traditional Chinese medicine, provide syndrome differentiation and holistic attendance, and effectively enhance the quality of life of elderly MHD sufferers from various aspects [5].

Auricular acupoint pressing bean method is an important therapy method in external therapy of traditional Chinese medicine, mainly through auricular acupoint pressing medicinal beans, regulating human endocrine, improving the function of abdominal organs, promoting blood circulation and removing blood stasis, etc., to enhance the symptoms of sufferers. Continued care is a part of overall care, that is, an extension of care, so that sufferers can receive continuous care during the recovery period during the entire therapy period [6]. The purpose of this paper is to provide a theoretical basis for the clinical care of MHD sufferers in the future.

RETRACTED

The rest of this paper is organized as follows: Section 2 discusses related work, followed by sufferers' information and intervention methods designed in Section 3.  Section 4 shows the experimental results and analysis. Finally, we sum up the research conclusion, point out the deficiencies, and propose the research direction for the subsequent studies in Section 5.

## 2. Related Work

When kidney disease develops to the end stage, in order to maintain the sufferer's life and prolong its survival time and cycle, it is necessary to replace the kidney with hemodialysis to remove metabolic waste from the body and maintain electrolyte and acid-base balance. However, over time, it will lead not only to immune dysfunction but also to inflammatory and hyperoxidative states, which will induce various complications. Therefore, there is a need to strengthen the intervention and implementation of effective care in therapy [7, 8].

The therapy concept of Chinese medicine is “disease prevention and mutation prevention.” The degree of hypertension depends on the number of sufferers undergoing hemodialysis. During dialysis, ultrafiltration is rapid and can notoriously reduce circulating blood pressure, induce hypotension, and cause muscle cramps [9]. Therefore, the most important part of routine care is to instruct sufferers to reduce fluid intake during dialysis and that body weight gain should not exceed 4%–5% dry matter. The usual therapy is the injection of calcium gluconate, but this therapy is not effective in sufferers after spastic attacks, the incidence of vascular calcification is higher in dialysis sufferers, and frequent injections of calcium gluconate can greatly increase the vascular. The risk of calcification, which Chinese medicine distinguishes as a whole, helps to enhance the sufferer's immune system [10]. Auricular point therapy is also a relatively common therapy method in Chinese medicine. Chinese medicine believes that there is a close relationship between the ear and the zang-fu meridians, and there are six yang meridians that circulate in and around the ear, respectively [11]. This examination found that the clinical efficacy of the sufferers in the examination set was notoriously higher than that in the contrast set, and the disparity was statistically extensive (*P* < 0.05), suggesting that it is feasible to apply auricular acupuncture in clinical therapy of diseases. Modern physiological studies have shown that the effects of auricular stimulation include multiple pathways. (1) The primary integration of information in the posterior horn of the spinal cord, thereby completing the intra-or intersegmental information reflex. (2) The somatosensory and visceral sensory nuclei in the brainstem. And (3) Information integration is carried out between the reticular nuclei in the reticular structure of the brainstem, and finally, the basic life activities of the body are adjusted [12, 13]. This examination found that after attendance, the TCM syndrome scores of the two sets of sufferers were decreased, and the examination set was notoriously lower than the contrast set (*P* < 0.05). BUN, SCr, and *β*2-M in the set were notoriously lower than those in the contrast set. Estimated glomerular filtration rate (eGFR) was notoriously higher than that in the contrast set, IL-6, IL-10, and hs-CRP in the two sets were decreased, and the examination set was notoriously lower than that in the contrast set (*P* < 0.05). For most elderly sufferers, they do not understand the related therapy of disease and MHD and due to the influence of disease pain and economic pressure during therapy, psychological pain and depression, and even loss of confidence in therapy, auricular acupuncture is applied to sufferers. After bean combined with continuous attendance, the quality of life of sufferers can be effectively enhanced in many aspects, and the implementation of emotional attendance can enhance the psychological state of sufferers and achieve the purpose of emotional peace and confidence, so as to actively cooperate with therapy [14]. Attendance can fully take care of the individual symptoms of elderly MHD sufferers, follow the constitution of traditional Chinese medicine, implement targeted therapy and dietary plans, and enhance the therapeutic effect. Ear acupoint pressing beans can effectively promote blood circulation, better sleep, and better relief Elderly MHD sufferers have various pains caused by complications and enhance the comfort of sufferers [15]. In conclusion, the implementation of auricular acupoint pressing beans + continuous attendance method has effectively and effectively enhanced the quality of life of sufferers.

RETRACTED

Chronic kidney disease is a major disease that threatens human health after tumors, seriously endangering the life and health of sufferers. MHD can effectively prolong life and enhance the quality of life. However, the elderly MHD sufferers are often accompanied by diabetes, hypertension, etc., which lead to complicated conditions, and MHD itself is also traumatic, causing sufferers to experience great physical and psychological pain during the therapy process [16]. This examination found that the follow-up time was until February 2022, and it was found that the readmission rate of the examination set was notoriously lower than that of the contrast set, and the survival rate was notoriously higher than that of the contrast set. The main reason for the decomposition is that auricular acupoint pressing beans combined with continuous attendance intervention have brought into play the characteristics of traditional Chinese medicine, people-oriented, relying on traditional Chinese medicine attendance techniques, and based on syndrome differentiation attendance and emotional conditioning to relieve sufferers' depression, pain, pain anxiety, so as to better intervene in the occurrence of complications in sufferers, give sufferers a better attendance experience, and enhance the physical pain and psychological pain of elderly MHD sufferers, so the sufferer's prognosis of readmission rate is notoriously reduced, and the prognosis of survival rate and quality of life are increased [17, 18]. Although this examination has achieved certain examination results, there are still limitations. Because only 110 sufferers were included in this examination, the sample size is small, which may cause certain biases in the results. Therefore, in the future examination, the sample size should be further expanded and further decomposition curative effect of auricular point pressing beans combined with continuous attendance on MHD.

## 3. Sufferers' Information and Intervention Methods

### 3.1. Sufferers' Information

In this examination, 110 elderly MHD sufferers who are treated in our hospital from February 2020 to February 2021 are selected as the examination objects, and they are randomly divided into two sets, 55 cases in the examination set and 55 cases in the contrast set. There are 30 males and 25 females in the examination set, the age range is 51–68 years old, the average age is (61.51 ± 4.21) years old, and the pathological types are as follows: polycystic kidney disease in 7 cases, chronic glomerulonephritis in 20 cases, diabetic nephropathy in 17 cases, and high 11 cases of hypertensive nephropathy. 32 cases of male and 23 cases of female in the contrast set, the age range is 50–69 years old, the average age is (61.59 ± 3.78) years old, the pathological types are as follows: 8 cases of polycystic kidney disease, 21 cases of chronic glomerulonephritis, 14 cases of diabetic nephropathy, 12 cases of hypertensive nephropathy. The general clinical data such as age, gender, and pathological type are in contrast between the two sets, *P* > 0.05, there is no extensive disparity between the two sets. All sufferers included in the examination signed the informed consent form. The therapy methods and detection methods applied in this examination are all known safe methods in the clinic. The general information and clinical data collected in this examination are only applied for examination decomposition, not for examination purposes. If you have any discomfort during the therapy, please inform your doctor in charge in time to decide on the next therapy plan. The entire therapy and observation period are 4 weeks, please inform the doctor of the changes in your condition in time, during the therapy, do not privately apply all other medicines and other therapies for this disease, and tell your doctor if you apply them.

RETRACTED

There are four inclusion criteria as follows: (1) Clear consciousness and no language, mental, or cognitive impairment. (2) Able to complete the questionnaire. (3) Diagnosed with chronic renal failure and MHD therapy for ≥ 12 months. (4) Sufferers voluntarily participated in this examination and signed an informed consent form.

There are two exclusion criteria as follows: (1) History of stroke, dementia, Parkinson's disease, and other neurological diseases. (2) Combined with stroke, severe heart failure, serious infection, malignant tumor, and other diseases.

### 3.2. Examination Methods

#### 3.2.1. Intervention Methods

All sufferers received routine hemodialysis therapy.

For the contrast set, the following intervention methods are implemented: Routine attendance is given to this set of sufferers, the urine output of the sufferers is monitored from time to time, and abnormal reactions such as anemia, edema, and electrolyte imbalance are closely observed.

For the examination set, the following intervention methods are implemented: The sufferers in this set are given auricular point pressing beans combined with continuous attendance intervention, the detailed methods are as follows: (1) Ear point pressing beans: the acupoint selection of this method mainly corresponds to the extensive intestine, rectum, and Sanjiao, and the corresponding spleen is selected for the sufferers according to the individual disparity of the sufferers, stomach, endocrine, sympathetic and other acupuncture points, as auxiliary points for sufferers. First, apply a carbon rod to identify and mark the positive acupoints of the sufferer's acupuncture points, then apply alcohol cotton balls to disinfect the sufferer's auricle, fix the sufferer's auricle with one hand, and apply the other hand to fix the sufferer's auricle. Apply tweezers to place the disposable Wangbuliuxing seed ear bean paste on the sufferer's ear acupuncture point and press it with fingers until the sufferer experiences soreness or slight pain, and instruct the sufferer and family members to press the area every day for 4∼5 times, press for about 3 minutes each time, and adjust the intensity of the pressing according to the sufferer's tolerance or dialectical needs, which can help enhance the overall therapeutic effect. Replace one side of the auricle every day for therapy. (2) Continuing attendance intervention: (1) Continuing attendance set: When implementing attendance intervention, the individual disparity of sufferers should be taken into account first, and attendance should be based on syndrome differentiation. The principle of balancing yin and yang is to formulate targeted and nutritious dietary recipes for elderly sufferers and urge sufferers to consume sufficient amounts of vitamins, iron, zinc, and other substances to enhance body tolerance and enhance prognosis. (2) Emotional conditioning: fully understand and evaluate their emotional state, and apply the method of soothing the mind and happiness, and the method of conquering emotions to regulate the sufferer's emotions and enhance the sufferer's mental health. (3) Acupoint massage: Experienced nurses provide training and guidance on acupoint massage for sufferers and their families. Massage Baihui, Neiguan, Yintang, Hegu, and other acupoints can effectively enhance sufferers' sleep. The massage time is 15–20 minutes. For sufferers with head pain, their family members can be instructed to learn the massage skills of the main acupoints on the head, such as Kan Palace, Tianmen, Fengfu, Bladder Meridian, and Shenting, and massage to relieve the headache. (4) Traditional Chinese medicine foot bath: guide the sufferer to take a traditional Chinese medicine foot bath before going to bed to enhance the blood circulation of the lower limbs and enhance the metabolism. The time of each foot bath should not exceed 30 minutes.

RETRACTED

#### 3.2.2. Serum and Renal Function Tests

In the morning fasting state, 5 ml of cubital venous blood is drawn from all participating examinations in the morning fasting state, centrifuged at 3 500 r/min for 10 min, the centrifugation radius is 10 cm, and serum Interleukin-6 (IL-6) is collected to be tested. Interleukin-10 (IL-10) and high-sensitivity C-reactive protein (hs-CRP). Blood urea nitrogen (BUN), serum creatinine (Scr), *β*2-microglobulin (*β*2-MG), and glomerular filtration rate are measured by the automatic biochemical resolver in the two sets of sufferers.

### 3.3. Observation Indicators

The observation indicators are as follows:

1. Contrast the clinical efficacy of the two sets [19], the criteria for clinical attendance effect: markedly effective is as follows: clinical symptoms disappeared completely, urine volume increased, and renal function notoriously enhanced. Effective: clinical symptoms are basically eliminated, urine volume increased, and renal function is notoriously enhanced enhancement. Ineffective is as follows: the sufferer's clinical symptoms, urine output, and renal function have all changed, or the disease has worsened. Total effective rate (%) = (marked number of people + effective number of people)/total number of people × 100%.
2. Comparing the enhancement of TCM symptom scores before and after attendance in the two sets. According to the Clinical Symptom Grading Quantitative Scale for sufferers with Uremia in the “Guidelines for Clinical examination of New Chinese Medicines in Treating Chronic Renal Failure” [20], the relevant symptoms are graded and quantified. Clinical symptoms are divided into main symptoms and secondary symptoms, which are divided into four grades: none, mild, moderate, and severe according to the degree, with 0, 1, 2, and 3 points, respectively. The scores of each sufferer are accumulated to obtain the TCM syndrome score of each sufferer. Before and after dialysis, the observation is recorded once, and the tongue and pulse are described in detail without scoring. There are five items including vomiting, stickiness in the mouth, poor appetite, abdominal distention, and physical distress, with scores ranging from 0 to 18. The higher the score, the worse the sufferer's condition.
3. The renal function indexes of BUN, SCr, *β*2-M, and eGFR are a contrast between the two sets of sufferers before and after attendance.
4. The expressions of IL-6, IL-10, and hs-CRP inflammatory factors are a contrast between the two sets before and after attendance.
5. Contrast of readmission and survival within one year of prognosis between the two sets.
6. The quality of life of the sufferers before and one year after attendance is a contrast between the two sets. The quality of life of the sufferers is assessed by the quality-of-life scale (WHOQOL-100) [21], which mainly includes the physical function, psychological function, and social function of the individual, substance survival status, and overall quality of life, using percentile scoring, 0–100 points, the higher the score, the better the quality of life.
7. To resolve the correlation between TCM symptom score and prognosis quality of life of sufferers.

RETRACTED

### 3.4. Statistical Methods

In this examination, all the data are organized, a corresponding database is established for it, all the databases are entered into SPSS 26.0 for data processing, and the measurement data is tested for normality, expressed as (*x* ± *s*), consistent with positive. The independent-sample *t* test is applied for the data between sets, the paired-sample *t* test is applied for the data within the set, and the Mann–Whitney *U* test is applied for non-normality. The rate is expressed as %, and the test is *χ*2. Correlation is resolved by Pearson. When *P* < 0.05, the disparity between the data is considered to be statistically extensive.

## 4. Experimental Results

### 4.1. Contrast of Clinical Efficacy between the Two Sets

Table 1 shows the contrast of clinical efficacy between the two sets. It can be seen from Table 1 that the clinical efficacy of the examination set is notoriously higher than that of the contrast set, and the disparity is statistically extensive (*P* < 0.05) after attendance.

### 4.2. The Enhancement of TCM Symptom Scores before and after Attendance in the Two Sets

Table 2 shows the contrast of TCM syndrome scores before and after attendance in the two sets. In Table 2, *∗*indicates that in contrast with before attendance, and *P* < 0.05, the disparity is statistically extensive. It can be seen from Table 2 that the TCM symptom scores of the two sets are higher, and the disparity is not statistically extensive (*P* > 0.05) before attendance. After attendance, the TCM syndrome scores of the two sets are decreased, and the examination set is notoriously lower than the contrast set (*P* < 0.05).

### 4.3. Contrast of Renal Function between the Two Sets of Sufferers before and after Attendance

Table 3 shows the contrast of renal function before and after attendance in the two sets of sufferers. In Table 3, *∗* indicates that in contrast with before attendance, and *P* < 0.05, the disparity is statistically extensive. It can be seen from Table 2 that there is no extensive disparity in renal function indexes of BUN, SCr, *β*2-M, and eGFR between the two sets (*P* > 0.05) before attendance. BUN, SCr, *β*2-M in the examination set are notoriously lower than those in the contrast set, and eGFR is notoriously higher than that in the contrast set, the disparity is statistically extensive (*P* < 0.05).

### 4.4. Contrast of Inflammatory Factors before and after Attendance in the Two Sets

Table 4 shows the contrast of inflammatory factors before and after attendance in the two sets. In Table 4, *∗* indicates that in contrast with before attendance, and *P* < 0.05, the disparity is statistically extensive. It is clearly evident from Table 4 that there is no extensive disparity in IL-6, IL-10, and hs-CRP inflammatory indexes between the two sets (*P* > 0.05) before attendance. All decreased, and the examination set is notoriously lower than the contrast set, the disparity is statistically extensive (*P* < 0.05).

RETRACTED

### 4.5. Prognosis of Readmission and Survival within One Year of the Two Sets

The follow-up time is until February 2022.  Table 5 shows the prognosis of readmission and survival within one year of the two sets.  Figure 1 shows the cumulative readmission rate within one year of prognosis in the two sets.  Figure 2 shows the cumulative survival rate within one year of prognosis in the two sets. Through the above experimental results, it can be observed that the readmission rate of the examination set is notoriously lower than that of the contrast set, the survival rate is notoriously higher than that of the contrast set, and the disparity is statistically extensive (*P* < 0.05).

### 4.6. Quality of Life before and One Year after Attendance in the Two Sets

Table 6 shows the contrast of the quality of life between the two sets at different time points. In Table 6, *∗* means contrast with before therapy, & means contrast with contrast set, and *P* < 0.05, the disparity is statistically extensive. It can be seen from Table 6 that the quality of life scores of the two sets are lower, and the disparity is not statistically extensive (*P* > 0.05) before intervention. After 1 year of therapy, the quality of life scores of the two sets are increased, and the examination set is notoriously higher than the contrast set (*P* < 0.05).

### 4.7. Correlation between TCM Symptom Score and Prognosis Quality of Life

The TCM syndrome scores and quality of life scores of the sufferers are collected.  Figure 3 shows the correlation between TCM symptom score and prognosis quality of life. It can be seen from Figure 3 that there is an extensive negative correlation between the two (*r* = −0.693, *P* < 0.001).

## 5. Conclusion

The effect of auricular point pressing beans + continuous intervention on *β*2-MG, curative effect, and its relationship with prognosis in elderly MHD sufferers is explored. For MHD sufferers, auricular acupuncture combined with continuous attendance during the therapy period can effectively enhance the clinical therapy effect, enhance the inflammatory index and renal function index, reduce the readmission rate, and enhance the prognosis quality of life, worthy of clinical application.

## Figures and Tables

**Figure 1:** Cumulative readmission rate within one year of prognosis in the two sets.

RETRACTED

**Figure 2:** The cumulative survival rate within one year of prognosis in the two sets.

**Figure 3:** Correlation between TCM symptom score and prognosis quality of life.

**Table 1:** Contrast of clinical efficacy between the two sets.

Set	Effective	Efficient	Invalid	Total efficiency
Contrast set (*n* = 55)	20 (36.36)	15 (27.27)	20 (36.36)	35 (63.64)
Examination set (*n* = 55)	35 (63.64)	15 (27.27)	5 (9.09)	50 (90.91)
*χ* ^*2*^				13.593
*P*				<0.001

**Table 2:** Contrast of TCM syndrome scores before and after attendance in the two sets.

Set	Before attendance	After attendance
Contrast set (*n* = 55)	13.56 ± 2.78	9.71 ± 2.38^*∗*^
Examination set (*n* = 55)	13.41 ± 2.59	5.36 ± 1.06^*∗*^
*t*	0.636	8.593
*P*	0.518	<0.001

**Table 3:** Contrast of renal function before and after attendance in the two sets of sufferers.

Set	BUN (mmol/L)		SCr (*μ*mol/L)		*β*2-M (mg/L)		eGFR (ml/min)	
	Before attendance	After attendance	Before attendance	After attendance	Before attendance	After attendance	Before attendance	After attendance
Contrast set (*n* = 55)	15.96 ± 3.82	11.25 ± 2.93^*∗*^	288.63 ± 76.51	268.97 ± 70.54^*∗*^	3.34 ± 1.92	2.69 ± 0.78^*∗*^	3.59 ± 0.63	5.62 ± 2.16^*∗*^
Examination set (*n* = 55)	15.49 ± 4.16	9.35 ± 2.13^*∗*^	295.61 ± 78.63	221.59 ± 70.51^*∗*^	3.41 ± 1.97	2.28 ± 0.63^*∗*^	3.62 ± 0.71	7.35 ± 2.41^*∗*^
*T*	0.653	11.528	0.781	12.351	0.569	9.527	0.396	10.563
*P*	0.529	<0.001	0.357	<0.001	0.627	<0.001	0.782	<0.001

**Table 4:** Contrast of inflammatory factors before and after attendance in the two sets.

Set	IL-6 (pg/L)		IL-10 (pg/L)		Hs-CRP (mg/L)	
	Before attendance	After attendance	Before attendance	After attendance	Before attendance	After attendance
Contrast set (*n* = 55)	147.85 ± 25.63	78.93 ± 11.77^*∗*^	133.52 ± 19.73	93.18 ± 10.43^*∗*^	19.86 ± 3.62	9.45 ± 1.27^*∗*^
Examination set (*n* = 55)	145.20 ± 23.57	67.89 ± 10.52^*∗*^	135.28 ± 20.15	71.52 ± 9.58^*∗*^	20.57 ± 3.49	5.16 ± 0.78^*∗*^
*T*	0.758	11.593	0.627	12.527	0.952	10.579
*P*	0.526	<0.001	0.681	<0.001	0.350	<0.001

**Table 5:** Prognosis of readmission and survival within one year of the two sets (*n*(%)).

Set	Readmission rate	Survival rate
Contrast set (*n* = 55)	19 (34.55)	51 (92.73)
Examination set (*n* = 55)	9 (16.36)	45 (81.82)
*χ* ^*2*^	12.563	16.571
*P*	<0.001	<0.001

**Table 6:** Contrast of the quality of life between the two sets at different time points.

Project	Set	Before therapy	1 year after therapy
The overall quality of life score	Examination set (*n* = 55)	72.31 ± 7.79	86.42 ± 6.38^*∗*^&
Project	Contrast set (*n* = 55)	69.81 ± 10.91	72.10 ± 7.35^*∗*^

## Data Availability

The simulation experiment data used to support the findings of this study are available from the corresponding author upon request.

RETRACTED

## References

[1] Wang M., Jiang H., He Q., Shi K., Liu H., Xue J. (2018). Effects of hemodialysis combined with hemoperfusion on renal function. *Micro-inflammatory State and Blood Purification in Sufferers with Chronic Renal Failure” Progress in Modern Biomedicine*.

[2] Zhou W. (2021). The application effect of ordinary hemodialysis and continuous hemodialysis in sufferers with chronic renal failure complicated with heart failure. *Dialysis and Artificial Organs*.

[3] Yang L. (2020). Effects of hemoperfusion combined with hemodialysis on micro-inflammatory state and renal function in sufferers with chronic renal failure. *Medical Journal of Chinese People’s Health*.

[4] Wang H. (2018). Clinical observation of female climacteric insomnia treated with auricular point pressing beans in combination with opening tianmen. *Henan Traditional Chinese Medicine*.

[5] Chen W. (2018). Curative effect and attendance strategies exploration of moxa box moxibustion combined with auricular point pressing with beans in the therapy of neck-shoulder and lumbocrural pains. *Chinese Journal of Convalescent Medicine*.

[6] Hu Q. (2019). Clinical examination on press-needle combined with auricular point pressing for hiccups after abdominal surgery. *New Chinese Medicine*.

[7] Chen L., Zhong Y., Xu Y., Zhang L., Xu D. (2019). Clinical examination on sishenwan tang combined with auricular point pressing with beans for diarrhea of yang deficiency of spleen and kidney type in ICU sufferers. *New Chinese Medicine*.

[8] Dong Q., Li T., Yu Y., Shen S. (2018). Clinical effect of auricular point pressing with beans in therapy of menopausal insomnia. *Nursing of Integrated Traditional Chinese and Western Medicine*.

[9] Yang W., Yan H., Pan Q. (2019). *Journal of Endocrinology*.

[10] Li H. (2022). Effect of psychological attendance intervention on the quality of life of elderly sufferers with uremia during maintenance hemodialysis. *Modern Digestive and Interventional Diagnosis and therapy*.

[11] Lv G., Zhang H., Kong L., Fan R., Huang L. (2020). Contrast of the incidence and influencing factors of falls in elderly and young and middle-aged maintenance hemodialysis sufferers. *Chinese Nursing Management*.

[12] Wang Y., Li Y., Chi Y., Zhang T., Wang B. (2021). The relationship between hemoglobin level and iron status evaluation indexes in elderly maintenance hemodialysis sufferers. *Shandong Medical Journal*.

[13] Zhang R., Guo J. (2020). Examination progress on psychological attendance of elderly maintenance hemodialysis sufferers. *Chinese Journal of Clinical Hepatology*.

RETRACTED

[14] Wang X., Yang M., Shen G. (2020). Effects of maintenance hemodialysis on cardiac structure and functional damage in elderly sufferers with renal failure. *Medical Journal of the Chinese People’s Armed Police Force*.

[15] Sun X., Chen R., Yu L. (2020). Application of three-dimensional integrated continuous attendance in maintenance hemodialysis sufferers with diabetic nephropathy. *Hainan Medical Journal*.

[16] Fang X., Zhang K., Wei Y., Wei X., Xu S., Li N. (2022). Intervention effect of painting art therapy on fatigue and sleep quality in young and middle-aged maintenance hemodialysis sufferers. *Chinese Journal of Practical Nursing*.

[17] Zhang C., Cai G. (2021). Research progress on prognostic factors in elderly hemodialysis patients. *Chinese Journal of Practical Internal Medicine*.

[18] Xia J., Song D., Zhu W., Zhou Y. (2021). Effect of exercise intervention during dialysis on the enhancement of quality of life and sleep quality in elderly maintenance hemodialysis sufferers under the multidisciplinary collaborative team model. *Practical Geriatrics*.

[19] Zeng B., Yang F. (2019). Curative effect of auricular point pressing bean combined with huatan tongmai therapy on stable Angina pectoris. *Chinese Journal of Integrative Medicine on Cardio-Cerebrovascular Disease*.

[20] Liu P., Zhang Z. (2019). Clinical observation on effect of auricular acupoint pressing with beans combined with point Application on postpartum milk secretion. *New Chinese Medicine*.

[21] He M., Wang E., Zhang L., Qiu Z., Miao S. (2019). Effect of continuous lumbar cistern drainage on intracranial pressure, complications and prognosis in elderly sufferers with severe craniocerebral injury. *Progress in Modern Biomedicine*.

